The article "Effect of Family Participatory Nursing Model Based on WeChat Platform on Psychological Elasticity and Quality of Life of Patients with Lung Cancer" was retracted in 2023. Reasons: signs of a paper mill; unreliable results or conclusions; concerns about the data; concerns about the results or conclusions.

# Effect of Family Participatory Nursing Model Based on WeChat Platform on Psychological Elasticity and Quality of Life of Patients with Lung Cancer

**DOI:** 10.1155/2022/4704107

**Published:** 2022-05-07

**Authors:** LingJuan Li, Fang Xu, Jun Ye

**Affiliations:** ^1^Department of Oncology, The First People's Hospital of Jingmen City, Hubei, China; ^2^Department of Respiratory, The First People's Hospital of Jingmen City, Hubei, China

## Abstract

**Objective:**

To explore the effect of family participatory nursing model based on WeChat platform on psychological elasticity and life quality of patients with lung cancer.

**Methods:**

One hundred patients with lung cancer treated in our hospital from February 2019 to April 2021 were enrolled. The patients were randomly assigned into control group and study group. The control group received routine nursing and the study group received family participatory nursing model based on WeChat platform. The scores of nursing satisfaction, self-feeling burden, symptom group assessment scale, family care index, and compliance and life quality were compared.

**Results:**

First of all, we compared the nursing satisfaction: the study group was very satisfied in 25 cases, satisfactory in 20 cases, general in 5 cases, the satisfaction rate was 100.00%; the control group was very satisfied in 14 cases, satisfactory in 17 cases, general in 13 cases, dissatisfied in 6 cases, and the satisfaction rate was 88.00%. Compared between the two groups, the nursing satisfaction in the study group was higher compared to the control group (*P* < 0.05). Secondly, we compared the self-perceived burden, the emotional burden, physical burden, and economic burden and total scores of the study group were lower compared to the control group (*P* < 0.05). Comparing the scores of symptom group evaluation scale, the scores of respiratory symptoms, fatigue symptoms, psychological and emotional symptoms, digestive tract symptoms, and nervous system symptoms in the study group were lower compared to the control group (*P* < 0.05). In terms of the family care index of the two groups, the scores of fitness, cooperation, length, emotion, and intimacy in the study group were higher compared to the control group (*P* < 0.05). Comparison of compliance, the study group was very compliant in 42 cases, compliant in 7 cases, noncompliant in 1 case, the compliance rate was 98.00%; the control group was very compliant in 24 cases, compliant in 20 cases, noncompliant in 6 cases, the compliance rate was 88.00%. The compliance rate in the study group was higher compared to the control group (*P* < 0.05). Finally, we compared the scores of qualities of life. Before nursing, there exhibited no significant difference (*P* > 0.05). The scores of physiological function, psychological function, social function, and health self-cognition in the study group were lower compared to the control group (*P* < 0.05).

**Conclusion:**

The family participatory nursing model based on WeChat platform helps to facilitate the psychological elasticity and quality of life of patients with lung cancer and further promote patients' self-care ability and compliance with lung cancer. It can also effectively enhance family care and nursing satisfaction; the nursing model is worth popularizing and applying in clinic.

## 1. Introduction

In the World Cancer Report-Cancer Prevention Research released by the International Cancer Institute of the World Health Organization (WHO) in 2020, global cancer statistics manifest that there will be an estimated 18.1 million new cancer cases and 9.6 million cancer deaths in 2018 [1]. The WHO counted 2.1 million new cases of lung cancer and 1.8 million deaths, accounting for 11.6% and 18.4% of the total number of cancers, respectively [2]. Globally, lung cancer is still the leading cause of cancerous morbidity and mortality. In China, according to the reports of the National Cancer Center in 2019, there are about 787,000 new cases of lung cancer every year, and the number of deaths from lung cancer is about 631,000 [3]. Cancer-related death is the leading cause of death in China [4]. Lung cancer accounts for 21.3% and 27.1% of the total morbidity and mortality of all kinds of cancers, respectively [5, 6]. The morbidity increases with age, and the mortality rate of males is higher compared to females, and the mortality rate of males is higher compared to females, and that of rural areas is higher compared to urban areas [7, 8]. Although the diagnosis and treatment of lung cancer are gradually standardized in our country, there is a lack of effective screening methods and most of the patients with early lung cancer have no significant symptoms, and most of the patients are diagnosed in the middle and late stage. The survival rate of population-based tumor registry in China indicates that during 2012-2015, the 5-year survival rate is 19.7% [9, 10].

At present, the treatments employed in the medical field are mainly surgery, supplemented by radiotherapy and chemotherapy [11]. Surgical treatment will cause inevitable trauma to the patient's body and then have a great impact on the patient's physiology and psychology [12]. During the period of hospitalization, patients with lung cancer will bear a variety of uncomfortable symptoms caused by diseases and treatment, and various symptoms occur, and the interaction increases the symptom burden of patients with lung cancer, thus affecting the treatment and prognosis [11, 12]. It is pointed out in the Code for diagnosis and treatment of Primary Lung Cancer (2015 Edition) that lobectomy is still the best choice for stage IA non-small-cell lung cancer (NSCLC) [13]. VATS is more widely employed in clinic, and the discomfort caused by the operation itself and various complications has become the main problem for medical staff. A variety of postoperative symptoms seriously affect the physical and mental health of patients, reduce patient satisfaction, and also reduce treatment compliance. In the actual medical work, patients may even lead to conflicts between doctors and patients because of wound pain, chest tightness, dyspnea, cough, and other reasons, so as to reduce the distress of postoperative symptoms to patients. Therefore, it is necessary for medical staff to objectively evaluate and effectively manage the postoperative symptoms. Although lung cancer patients have won a longer life period after operation, radiotherapy, and chemotherapy, they have paid the price of reducing the quality of life [14]. After the patients receive treatment, conventional nursing cannot achieve effective results, so it is necessary to find a new nursing model.

The Family Participatory Care model, which emphasizes the involvement of the patient's family in the whole process of care during the rehabilitation process, was first introduced in China in 2016 [15]. It is mostly employed in the nursing of premature infants, but there are few reports on clinical nursing of patients with lung cancer. WeChat, as a new media, has gradually appeared in various fields. As a new way of social interaction, WeChat has the characteristics of convenient, fast, timely, dynamic, and continuous [15]. The survey indicates that the coverage rate of WeChat users in Chinese big cities has reached 92.6%. The family participatory nursing model based on WeChat platform can not only realize remote rehabilitation guidance but also dynamically grasp the rehabilitation process of patients and give targeted nursing guidance, and the family members of patients can participate in the rehabilitation nursing process throughout the process. It can not only facilitate the nursing skills of family members but also help to urge patients to cooperate actively [16]. Therefore, this study explores the impact of WeChat-based family participatory nursing model on the psychological elasticity and life quality of patients with lung cancer, in order to provide empirical basis for rehabilitation management of lung cancer.

## 2. Patients and Methods

### 2.1. General Information

One hundred patients with lung cancer treated in our hospital from February 2019 to April 2021 were enrolled. The patients were randomly assigned into control group and study group. The control group received routine nursing and the study group received family participatory nursing model based on WeChat platform. In the control group, the age was 35-74 years old, with an average age of 50.64 ± 3.44 years, containing 23 males and 27 females, while in the study group, the age was 34-76 years old, with an average age of 50.77 ± 3.44 years, containing 26 males and 24 females. There was no statistical significance in the general data of the two groups. This study was permitted by the Medical Ethics Association of our hospital, and all patients signed informed consent.

Inclusion criteria are as follows: (1) patients undergoing thoracoscopic lung cancer surgery (confirmed by clinical and histopathology); (2) age ≥ 18 years old; (3) patients without other cancers; (4) disease permission, willing to cooperate with the investigation; (5) clear consciousness, no cognitive dysfunction and communication disorders; and (6) informed consent of the patients.

Exclusion criteria are as follows: (1) patients with poor general condition, i.e., the heart, lung, liver, kidney, and other important organ functions unable to tolerate the operation; (2) preoperative movement disorder; (3) patients with active bleeding tendency after operation; (4) diagnosed stage IV, most of stage III B and part of stage III A NSCLC; and (5) patients who changed from thoracoscopic surgery to thoracotomy.

### 2.2. Treatment Methods

The control group received routine nursing intervention in the department, issued the disease guidance manual to the patients on the day of admission, evaluated the admission, patiently carried out health education for the patients, and explained to the patients the matters needing attention in disease-related self-management. Individualized nursing guidance is given, and the way of education is mainly through health education. Instruct the patients to breathe through the abdomen, draw the lips, blow balloons, and climb stairs one day before operation, and explain to the patients the mode of operation, the time of fasting water, the preparation of patients before operation, and the purpose of medication before operation. Postoperative matters need attentions, such as postoperative drinking time, diet education, postoperative posture, and time to get out of bed. Discharge health education includes hospital review a week later, revisit at any time when the condition changes, pay attention to keep warm, avoid catching cold and going to crowded places, and eat a diet high in protein, high in vitamins, light and easy to digest, and avoid drinking alcohol within a week.

The research group accepted the family participatory nursing model based on WeChat platform: the members of the group included 1 oncologist (deputy chief physician), 1 nursing expert (chief nurse), 1 psychological counselor, 1 specialist nurse (nurse), and 1 WeChat instructor (researcher himself). Doctors are responsible for explaining and guiding the knowledge of lung cancer-related diseases and supervising the whole intervention process; psychological counselors guide conversation methods; nursing experts and specialist nurses participate in the development of health guidance manuals for lung cancer patients; the researcher is responsible for sending WeChat intervention programs and supervising the whole WeChat intervention process. On the day of admission, the researchers added WeChat with the patient's family, established a WeChat group named “patient group”, and invited family participation group members to join the group to confirm that family members and patients joined the group by scanning QR codes. On the second day after discharge, the researchers began to send information to the patients' families, containing basic knowledge of lung cancer, knowledge of self-care, rehabilitation training methods, and daily life guidance through WeChat voice or video to urge patients' families to convey the effect of self-care in a timely manner and guide patients to conduct rehabilitation training on time. The patients and their families reported the situation at home to the researchers every week, containing whether the rehabilitation training was carried out correctly.

#### 2.2.1. Observation Index

*(1) Satisfaction*. After consulting the literature and experts' discussion, we designed patients' follow-up satisfaction, a total of 10 items, and recorded patients' satisfaction with follow-up management mode, health education, medical and nursing service, appointment registration process, and so on [17]. It is assigned into four dimensions: very satisfied, satisfied, general, and dissatisfied. Satisfaction rate = very satisfaction rate + satisfaction rate + general rate.

#### 2.2.2. Self-Perceived Burden Score

Self-perceived burden scale (SPBS), the scale includes three dimensions, a total of 10 items [18], that is, physical burden (1, 2, 5, 7, 8), emotional burden (4, 6, 9, 10), and economic burden (3). The scale was scored by the Likert 5 grade, with 5 points for “always”, 4 points for “often”, 3 points for “sometimes”, 2 points for “occasionally” and 1 point for “no”. According to the score of SPB, it can be assigned into >40 points as severe self-feeling burden, 30 points ≤ SPB<40 points as moderate self-feeling burden, 20 points ≤ SPB<30 points as mild self-feeling burden, and<20 points as no obvious self-feeling burden. The total score of the scale ranged from 10 to 50, and the higher the score, the heavier the burden. Cronbach's *α* coefficient of this study is 0.85.

#### 2.2.3. Symptom Group Assessment Scale

The Chinese version of the Anderson symptom Assessment scale (MDASI-C), the revised MDASI-C consists of three parts [19]. The first part assesses the severity of 13 common symptoms of cancer, such as drowsiness, fatigue, and pain, within 24 hours, with each score from 0 to 10, representing the range from “asymptomatic” to “the most severe imaginable”. The second part evaluates the effects of the above 13 symptoms on six aspects of daily life, such as walking, work, and relationships with others. Each item uses a scoring method similar to that of the first part, from 0 to 10 points, which represents from “non-interference” to “complete interference”. The third part is the specific symptoms of lung cancer, which evaluates the severity of cough, expectoration, hemoptysis, chest tightness, constipation, and weight loss in the past 24 hours, from 0 to 10 points. It represents that from “no symptom” to “the symptom reached the most severe degree”, the score is proportional to the severity of the symptoms. Cronbach's *α* coefficient of the revised MDASI-C scale was 0.925. Cronbach's *α* coefficient of this study is 0.80.

#### 2.2.4. Family Care Index

Family Care Index questionnaire is assigned into five items corresponding to five dimensions, namely, family fitness, cooperation, length, emotion, and intimacy [20]. The questionnaire was scored with 3 grades, 0 for almost nothing, 1 for sometimes, and 2 for frequent, and the final score was the sum of 5 dimensions. The higher the score, the better the family function. Cronbach's *α* coefficient is 0.89.

*(1) Compliance*. Statistics on the compliance of the two groups of patients are very compliant: patients completely follow the guidance of medical staff, can take medicine regularly, and conduct self-care and self-rehabilitation. In compliance, most of the patients follow the guidance of medical staff. Most of the time, they can take medicine regularly and conduct self-care and self-rehabilitation. In noncompliance, patients do not fully follow the guidance of medical staff, who cannot use medicine regularly and conduct self-care and self-recovery. Compliance rate = very compliance rate + compliance rate.

#### 2.2.5. Life Quality Scale

The life quality scale consists of four subscales, containing physical, psychological, social, and health self-awareness with a total of 29 items [21]. Cronbach's *α* coefficient of the scale is 0.79 to 0.91. The scale was scored by 1-5 grades. The lower the score, the higher the satisfaction.

### 2.3. Statistical Analysis

Two-person input data employed the SPSS21.0 statistical software package under the guidance of statistical experts for statistical analysis. Frequency, constituent ratio, and standard deviation were employed to describe the statistical data; chi-square test was employed for general data; rank sum test was employed for intergroup comparison and two-sample comparison. The data were tested by bilateral test, and the test level *α* was set to 0.05 (*P* < 0.05), which indicated that the difference exhibited statistical significance.

## 3. Results

### 3.1. Comparison of Nursing Satisfaction

First of all, we compared the nursing satisfaction: the study group was very satisfied in 25 cases, satisfactory in 20 cases, general in 5 cases, the satisfaction rate was 100.00%; the control group was very satisfied in 14 cases, satisfactory in 17 cases, general in 13 cases, dissatisfied in 6 cases, and the satisfaction rate was 88.00%. The nursing satisfaction in the study group was higher compared to the control group (*P* < 0.05). All the data results are indicated in Figure 1.

### 3.2. Comparison of Self-Perceived Burden

Secondly, we compared the self-perceived burden, the emotional burden, physical burden, and economic burden and total scores of the study group were lower compared to the control group (*P* < 0.05). All the data results are indicated in Table 1.

### 3.3. Comparison of Symptom Group Assessment Scale

Thirdly, we compared the scores of symptom group evaluation scale. The scores of respiratory symptom group, fatigue symptom group, psychological and emotional symptom group, digestive tract symptom group, and nervous system symptom group in the study group were lower compared to the control group (*P* < 0.05). All the data results are indicated in Table 2.

### 3.4. Comparison of Family Care Index

Then, we compared the family care index. The scores of fitness, cooperation, length, emotion, and intimacy in the study group were higher compared to the control group (*P* < 0.05). All the data results are indicated in Table 3.

### 3.5. Compliance Comparison

Next, we compared the compliance: the study group was very compliant in 42 cases, compliant in 7 cases, and noncompliant in 1 case, with a compliance rate of 98.00%; the control group was very compliant in 24 cases, compliant in 20 cases, and noncompliant in 6 cases, and the compliance rate was 88.00%. The compliance rate in the study group was higher compared to the control group (*P* < 0.05). All the data results are indicated in Figure 2.

### 3.6. Comparison of the Qualities of Life Scores

Finally, we compared the scores of qualities of life. Before nursing, there exhibited no significant difference (*P* > 0.05). The scores of physiological function, psychological function, social function, and health self-cognition in the study group were lower compared to the control group (*P* < 0.05). All the data results are indicated in Table 4.

## 4. Discussion

Lung cancer is the most common lung malignant tumor [22]. According to the cancer statistical report released by the World Health Organization International Cancer Research (IARC) in 2021, there are about 19.29 million new cancer cases and 9.95 million deaths in the world in 2020. Among them, the number of new cases of lung cancer in 2020 was about 2.2 million, and the number of deaths was about 1.79 million. Lung cancer ranks second in new cases of cancer and ranks first in cancer deaths [22]. In China, lung cancer is the first malignant tumor in morbidity and mortality. In 2020, the number of new cases of lung cancer is about 810 thousand, and the number of deaths is about 710 thousand [21, 22]. The incidence of lung cancer is relatively hidden, most patients are already in the advanced stage at the time of diagnosis [23], of which 57% of the patients have distant metastasis. The prognosis of patients with advanced lung cancer is often poor, and the 5-year survival rate of patients with stage IV lung cancer is only 6%. Studies have indicated that patients with advanced lung cancer have a lower life quality than other cancers. Life quality is not only an evaluation index to reflect the individual's perceived physical, psychological, and social adaptation to life but also an important predictive index to evaluate the survival time of patients [21]. Being diagnosed with cancer not only affects the physical and mental health of the patient but can also place a psychological and physical burden on them. In addition, advanced lung cancer has a lower life quality than caregivers of patients with other chronic diseases. Therefore, in the process of cancer management, the view of “focusing on the patient's disease participation while ignoring the patient's psychological and social function” is out of date [24]. More scholars encourage to regard cancer as a stressful event involving patients. Previous studies have confirmed that in the whole process of cancer treatment, patients have an interdependent relationship between physiology and psychology, which influence each other.

Psychological resilience is the internal coping resources available to the individual, and it is a kind of ability and character that the individual has [25]. Psychological resilience refers to the individual's ability to recover and adapt well from adversity, major traumatic and threatening events. When individuals are faced with stressful events and adversity, psychological resilience can help them strengthen their ability to deal with stressful events, reduce the mental blow caused by this event, promote the process of adaptation, and facilitate the quality of life of individuals [25]. Resilience has become a hot topic in the field of cancer. Previous studies have proved that resilience can protect individuals from the side effects of negative events and reduce the shock of cancer diagnosis [25, 26]. Among cancer patients, psychological resilience is thought to be associated with better disease adaptation and clinical outcomes and a higher life quality. A study of cancer patients receiving hematopoietic stem cell transplantation demonstrated that patients with high psychological resilience reported better physical, psychological, and social functions and life quality than patients with low psychological resilience [26]. In another study of elderly cancer survivors (over 65 years old), it was found that survivors with higher psychological resilience had better physical function [27]. Some scholars have studied 970 patients with digestive tract cancer. The results manifest that psychological elasticity can facilitate the life quality of patients by reducing the symptoms of physical fatigue and psychological disturbance caused by treatment. In the study of patients with early breast cancer, some scholars found that patients with low psychological elasticity at baseline had higher psychological pain and worse psychosocial adaptability after 6 years. There was a significant negative correlation between psychological pain and poor psychosocial adaptability and life quality [28]. Some studies have also found that high psychological resilience can promote patients' adaptation to the disease, strengthen their coping ability, reduce anxiety and depression, and facilitate their life quality. A study on caregivers of cancer survivors also found that psychological resilience can help patients better cope with stress and adapt to the new environment, and patients with high psychological resilience have less self-burden and psychological distress and a higher life quality [28]. Xu found that a high level of psychological elasticity can reduce the harmful effects of stress events on patients, making patients become more optimistic and experience less burden and helplessness, which plays a positive role in promoting the life quality of patients [29].

The participation and support of family members is very important to the rehabilitation of patients with lung cancer, and good family function plays a vital role in the physical and mental development of individuals [29]. The family care index includes five dimensions: fitness, cooperation, length, emotion, and intimacy. Fitness refers to the ability of individuals to use family resources to solve problems when they encounter difficulties; cooperation refers to the degree of shared responsibility of family members; growth length refers to the degree to which individuals are supported by family members; emotional degree refers to the degree of mutual care among family members; intimacy refers to the degree of sharing of time and money among family members. Our study demonstrated that regarding the family care index of the two groups, the scores of fitness, cooperation, length, emotion, and intimacy in the study group were higher compared to the control group. It indicates that the family participatory nursing model based on WeChat platform can obviously facilitate the family function. The reason may be as follows: first of all, this study sends relevant rehabilitation knowledge through WeChat platform and regularly urges family members to actively participate in the rehabilitation process of patients, which is beneficial to help family members maintain correct disease awareness, and family members talk to patients regularly. Understanding the psychological needs and expectations of patients helps to increase the understanding and acceptance of patients by family members, giving care and support to patients and maintaining good family relationships. Secondly, through the WeChat group, the contact between patients' families and medical, nursing, and psychological experts is strengthened, and the experts timely and accurately correct improper rehabilitation training methods, which is conducive to giving full play to the subjective initiative of patients and their families, obtaining the cooperation of family members and increasing patients' confidence in active rehabilitation. Finally, the family participatory care model based on the WeChat platform focuses on strengthening the synchronization of the patient's family members in the rehabilitation process, providing feedback on relevant issues through the WeChat platform to promote effective patient self-care and rehabilitation.

In terms of the results of this study, the nursing satisfaction of the two groups was compared: the study group was very satisfied in 25 cases, satisfactory in 20 cases, general in 5 cases, the satisfaction rate was 100.00%; the control group was very satisfied in 14 cases, satisfactory in 17 cases, general in 13 cases, dissatisfied in 6 cases, the satisfaction rate was 88.00%. The nursing satisfaction in the study group was higher compared to the control group. In the comparison of self-perceived burden, the scores of emotional burden, physical burden, economic burden, and total burden in the study group were lower compared to the control group. Comparing the scores of the symptom group evaluation scale, the scores of respiratory symptoms, fatigue symptoms, psychological and emotional symptoms, digestive tract symptoms, and nervous system symptoms in the study group were lower compared to the control group (*P* < 0.05). The scores of qualities of life of the two groups were compared. Before nursing, there exhibited no significant difference (*P* > 0.05). The scores of physiological function, psychological function, social function, and health self-cognition in the study group were lower compared to the control group (*P* < 0.05). The analysis indicates the following: first of all, the family members are included in the whole process of rehabilitation care of lung cancer patients through WeChat platform, and the rehabilitation plan is directly sent to the patients' family members by WeChat video or voice text, and the family members learn and master skills step by step, fully understand the language information, and increase the communication time with patients. Secondly, through the close contact with the patient's family, the patient's family's trust in the medical staff is enhanced, the rehabilitation method is brought back to the family quickly and efficiently from the hospital, and the hospital and family integration is realized. It ensures the continuity, integrity, and sustainability of the rehabilitation process. Finally, experts give targeted online guidance to the problem, family members quickly and efficiently master and effectively urge patients to conduct self-rehabilitation at home, which is helpful to facilitate the living ability of patients. Comparison of compliance between the two groups, the study group was very compliant in 42 cases, compliant in 7 cases, noncompliant in 1 case, the compliance rate was 98.00%; the control group was very compliant in 24 cases, compliant in 20 cases, noncompliant in 6 cases, the compliance rate was 88.00%. The compliance rate in the study group was higher compared to the control group. The analysis indicates the following: first of all, the family participatory nursing model based on WeChat platform allows patients to learn health data related to lung cancer and appropriately master the relevant knowledge of self-care of lung cancer through telephone return visit; secondly, the research group establishes contact with the family members of patients through the WeChat platform, which is convenient to provide correct guidance to the family members, and can more intuitively understand the disease-related knowledge. Finally, in the process of intervention, the family members of the patients were assessed through the WeChat platform, which helps to strength the family members' mastery of disease-related knowledge.

## 5. Conclusions

Conclusively, the family participatory nursing model based on WeChat platform helps to facilitate the psychological elasticity and quality of life of patients with lung cancer and further promote facilitating patients' self-care ability and compliance with lung cancer. It can also effectively enhance and facilitate family care and nursing satisfaction, the nursing model is worth popularizing and applying in clinic.

## Figures and Tables

**Figure 1:** Comparison of nursing satisfaction between two groups.

**Figure 2:** Comparison of compliance between two groups of patients.

**Table 1:** Comparison of self-perceived burden between the two groups [$\bar{x}\pm s$, Points].

Group	*N*	Emotional burden	Physical burden	Economic burden	Total burden score
C group	50	12.38 ± 2.34	15.69 ± 1.22	3.42 ± 1.24	30.82 ± 2.11
R group	50	8.22 ± 0.55	11.26 ± 4.21	2.35 ± 2.44	21.56 ± 2.55
*t*		12.237	7.146	2.764	19.783
*P*		<0.01	<0.01	<0.01	<0.01

**Table 2:** Comparison of the scores of symptom group assessment scale between the two groups [$\bar{x}\pm s$, Points].

Group	*N*	Respiratory symptom group	Fatigue symptom group	Psychological and emotional symptom group	Digestive tract symptom group	Nervous system symptom group
C group	50	2.58 ± 0.54	3.55 ± 0.31	1.84 ± 0.07	1.48 ± 0.51	1.93 ± 0.12
R group	50	1.93 ± 0.33	1.58 ± 0.12	1.07 ± 0.45	1.04 ± 0.43	1.06 ± 0.33
*t*		7.262	41.905	11.955	4.663	17.519
*P*		<0.01	<0.01	<0.01	<0.01	<0.01

**Table 3:** Comparison of family care index between the two groups [$\bar{x}\pm s$, Points].

Group	*N*	Fitness degree	Cooperation degree	Into length	Emotional degree	Intimacy
C group	50	1.24 ± 0.42	1.39 ± 0.57	1.44 ± 0.67	1.34 ± 0.56	1.45 ± 0.55
R group	50	2.06 ± 0.84	2.23 ± 0.42	2.52 ± 0.31	2.22 ± 0.31	2.21 ± 0.45
*t*		6.173	8.389	10.344	9.721	7.562
*P*		<0.01	<0.01	<0.01	<0.01	<0.01

**Table 4:** Comparison of quality-of-life scores between the two groups before treatment [$\bar{x}\pm s$, Points].

Group	*N*	Physiological function		Psychological function		Social function		Healthy self-cognition	
		Before nursing	After nursing	Before nursing	After nursing	Before nursing	After nursing	Before nursing	After nursing
C group	50	15.30 ± 4.42	13.86 ± 2.44a	16.42 ± 3.65	14.32 ± 4.76a	18.21 ± 3.53	16.49 ± 2.67a	15.67 ± 3.44	13.76 ± 1.34a
R group	50	15.53 ± 4.75	10.84 ± 2.91b	16.55 ± 3.46	12.44 ± 1.42b	18.71 ± 3.86	12.81 ± 3.54b	15.76 ± 3.34	10.12 ± 2.77b
*t*		0.250	5.623	0.182	2.676	0.675	5.868	0.132	8.364
*P*		>0.05	<0.01	>0.05	<0.01	>0.05	<0.01	>0.05	<0.01

Note: the control group before and after nursing, aP < 0.05; the study group before and after nursing, bP < 0.05.

## Data Availability

All the data involved in this study have been included within the article.
